This article has been retracted.

# Rituximab May Have Positive Effect on Refractory Nephrotic Syndrome: A Meta-Analysis of Randomized Trials

**DOI:** 10.1155/2022/3008597

**Published:** 2022-06-30

**Authors:** Jingjing Lin, Jia Sun

**Affiliations:** Nephrology Department, First People's Hospital of Linping District, Hangzhou, China

## Abstract

**Purpose:**

This study was aimed at demonstrating the role of rituximab (RTX) on the influence of nephrotic syndrome (NS) and on urinary protein which was not significant.

**Methods:**

The clinical randomized controlled trials were performed by eight databases. Meanwhile, the confidence interval (CI) of either relative risk or mean difference was set to 95%. Besides, the heterogeneity of the research results is tested by *I*^2^.

**Results:**

A total of 1658 references were found using the search method. This meta-analysis will be done by the ultimately eight different studies. Each study is described as random controlled trial. According to these eight studies, the remission of test group and control group was quite higher (OR: 1.60; 95% Cl: 1.17, 2.20; *P* < 0.01) than the control group, serum albumin (SMD: 4.19; 95% Cl: 1.49, 6.89; *P* < 0.01), and urine protein (SMD: 0.79; 95% Cl: -0.64, 2.22; *P* = 0.28). Despite the fact that the remission rate's funnel plot was asymmetrically distributed, Egger's test and Begg's test revealed no probable publish bias.

**Conclusion:**

The results of this study suggest that rituximab (RTX) may be effective in RNS, as evidenced by remission rates and serum albumin. However, the effect on urinary protein was not significant. The clear evidence is missing in this literature. Therefore, large sample, multicenter, low risk of bias clinical studies, as well as basic medical research, is needed.

## 1. Introduction

Severe proteinuria and episodes of hypoproteinaemia (serum albumin 2.5 g/dl) characterized nephrotic syndrome (NS), which is frequently linked with dyslipidaemia and hypercoagulability. Focal segmental glomerulosclerosis is usually resistant to corticosteroids and had a higher risk of kidney failure, needing renal transplantation. The disease affects 2-10 children per 100,000 people per year in western countries, with a prevalence of 16 cases per 100,000 people [1]. Different genetic and clinical variants are involved in the disease's underlying mechanisms [2, 3], with polymorphic podocyte destruction serving as a unifying feature [4, 5]. From minor lesions (minimal change disease) to podocyte depletion and glomerulosclerosis, all of the symptoms described are considered part of a pathology continuum (focal and segmental glomerular sclerosis) [4].

Oral corticosteroids are the cornerstone of treatment, with 90 percent of patients experiencing remission [6–8]. However, up to 85% of these individuals relapse within 5 years, and many acquire a steroid dependency [9, 10]. In such situations, the condition recurs within two weeks of quitting the steroids, necessitating the continuation of treatment indefinitely. Alternative therapy alternatives must be sought due to the toxicity of these drugs [11].

Rituximab (RTX) is a genetically produced chimeric murine/human monoclonal antibody that inhibits B cell proliferation and differentiation by targeting the CD20 antigen on the surface of B cells. It inhibits B lymphocyte proliferation and differentiation by targeting the CD20 antigen on their surface. RTX was first used in clinical practice to treat non-Hodgkin's lymphoma; subsequently, it was broadened to include autoimmune diseases [12]. RTX has been demonstrated to be beneficial in maintaining remission in refractory NS (RNS) in recent uncontrolled studies [13]. Thus, we conducted a meta-analysis to examine the association between RTX and RNS in the hope of providing a reference for the formulation and practice of RNS.

## 2. Materials and Methods

### 2.1. Inclusion Criteria

Articles that meet the conditions of population, intervention, comparators, outcomes, and study (PICOS) design were included into this study.

### 2.2. Exclusion Criteria

(1) Nonrandomized controlled trial research literature, (2) literature that did not report RTX as an intervention measure, (3) literature without original data or incomplete research data; (4) inconsistent outcome indicators or statistical methods; and (5) literature review or animal experiment research.

### 2.3. Design of the Research

All randomized controlled trials (RCTs) investigating RTX combined with other therapies in the treatment of RNS were not limited by language or publication status.

### 2.4. Research Object

Inclusion of patients with RNS, including hormone resistant NS, hormone-dependent NS, and patients with frequent recurrent NS.

### 2.5. Intervention Measures

The experimental group received RXT or RTX in combination with other medications for intervention, whereas the control group received non-RTX treatments such as hormone or immunosuppressive therapy. Furthermore, the two groups received treatment at the same time. Studies that did not match all of the criteria for inclusion were eliminated.

### 2.6. Outcome Indicators

The researcher discovered that the most widely used evaluation indicators for RNS are remission rate, serum albumin, and urine protein after reviewing clinical trials published in major databases and academic journals. The remission rate of the test and control groups was reported in eight investigations. The serum albumin of the test and control groups was reported in four investigations. The blood albumin of the test and control groups was reported in previous studies.

### 2.7. Search Strategy

This is a search method. Up until March 2022, we searched PubMed, Embase, Cochrane Library, Web of Science, CNKI, VIP, WanFang, and CBM Libraries for relevant randomized controlled trials. For English databases, we used free text terms such as “rituximab” or “refractory nephrotic syndrome”.

### 2.8. Literature Screening and Data Extraction

Two researchers independently conducted literature screening in strict conformity with inclusion and exclusion criteria and used NoteExpress software to manage and identify the retrieved material. After picking, researchers read the topic and abstract for preliminary screening and then further read the full text for rescreening to determine whether to include and extract valid data, respectively, to establish Excel effective data extraction table. In case of disagreement, a third researcher shall be invited to solve the disagreement through consultation.

### 2.9. Statistical Analysis

Stata 15.1 software was used to perform the meta-analysis. If for the binary classification variables using relative risk (RR), the confidence interval (CI) is set to 95%. Continuity variables were represented by mean difference (MD), and confidence interval (CI) was set at 95%. Heterogeneity of research results was tested by *I*^2^. If *I*^2^ ≤ 50%, outcome data of fixed effects model (FE) were selected for analysis; if *I*^2^ > 50%, outcome data of random effects model (RE) were selected for reference analysis. At the same time, sensitivity analysis was used to observe heterogeneous sources and evaluate the stability of meta-analysis results.

## 3. Results

### 3.1. Search Results

A total of 1658 references were found using the search method. After removing duplicate research, the abstracts and titles of 825 studies were scanned. The whole text of 43 articles was then reviewed. Following a full manuscript review, ten records were eliminated for the following reasons, of which 18 were not RCT and 7 had no outcomes. This meta-analysis eventually included 8 studies [14–21] (Table 1). This method is depicted in the PRISMA statement flow chart (Figure 1).

### 3.2. Remission Rate

The remission rate of the test and control groups was reported in eight investigations [14–21]. The test group's remission rate was substantially lower (OR: 1.44; 95 percent Cl: 0.99, 2.12; *P* = 0.059; *I*^2^ = 79.6 percent, Figure 2) than the control group (OR: 1.44; 95 percent Cl: 0.99, 2.12; *P* = 0.059; *I*^2^ = 79.6 percent, Figure 2). Because the findings of all of these trials were highly heterogeneous, a sensitivity analysis was performed (Figure 3), which revealed that the included trials [20] had a greater impact on the outcomes. According to the included article, the route originated in China. After excluding this trial, the remaining 7 studies were used to get new result (OR: 1.60; 95% Cl: 1.17, 2.20; *P* < 0.01; *I*^2^ = 58.2%, Figure 4). Heterogeneity decreased compared to the previous results, and excluded trials were consistent with sensitivity analysis results.

### 3.3. Serum Albumin

The serum albumin of the test and control groups was reported in four investigations [14, 16, 18, 20]. The serum albumin of the test group was considerably greater than the control group (SMD: 4.19; 95% Cl: 1.49, 6.89; *P* < 0.01; *I*^2^ = 99.8%, Figure 5) according to a meta-analysis.

### 3.4. Urine Protein

The blood albumin of the test and control groups was reported in three studies [14, 16, 18, 20]. The serum albumin of the test group was substantially greater (SMD: 0.79; 95 percent Cl: -0.64, 2.22; *P* = 0.28; *I*^2^ = 99.3 percent, Figure 6) than that of the control group (SMD: 0.79; 95 percent Cl: -0.64, 2.22; *P* = 0.28; *I*^2^ = 99.3 percent, Figure 6).

### 3.5. Publication Bias

Despite the fact that the remission rate's funnel plot (Figure 7) was asymmetrically distributed, Egger's test (*P* = 0.293) and Begg's test (*P* = 0.266) revealed no probable publish bias.

## 4. Discussion

NS is a group of syndromes with similar clinical manifestations due to multiple etiologies. It is typically characterized as profuse proteinuria, high oedema, hyperlipidaemia, and hypoproteinaemia. Hormone therapy was once widely used; however, a small percentage of individuals with nephrotic syndrome were found to be resistive to microscopic nephrotic syndrome following withdrawal of hormone therapy.

The exact cause of nephrotic syndrome is uncertain; however, immunological disorders mediated by T cells are considered to play a role [22]. B cells have been demonstrated to increase T cell activation, mediate antibody-independent autoimmune damage, and offer costimulatory substrates and cellular factors that keep T cells active in autoimmune disorders in several studies [23, 24]. Rituximab reduces B cell multiplication and causes apoptosis in B cells. This treatment causes B cell depletion, which prevents nephrotic syndrome recurrence by limiting the interaction between B cells and T cells. In patients with marginally changed nephrotic syndrome, impaired regulatory T cell function and regulatory T cell-induced nephrotic syndrome remission have previously been observed [25]. The drug rituximab boosts the number and function of regulatory T cells. The restoration of regulatory T cell function may be the reason for rituximab-maintained nephrotic syndrome remission.

This study showed that patients with RNS who received RTX had higher remission rates compared with controls. Meta-analysis showed satisfactory remission rates for RTX for RNS (OR: 1.60; 95% Cl: 1.17, 2.20; *P* < 0.01). The stability of the results was high after removing a trial with high heterogeneity. RXT significantly enhanced serum albumin levels in RNS patients compared to controls, according to the results of a meta-analysis of serum albumin levels (SMD: 4.19; 95 percent Cl: 1.49, 6.89; *P* < 0.01). However, there was no statistical difference in urine protein levels between the control and observation groups following treatment with RTX.

This study also has certain disadvantages. First, there are about 8 RCTs including 459 patients. The overall sample size is not very large. All RCTs were single-center. The lack of multicenter studies may affect the representativeness of the conclusions to some extent. Second, the primary outcomes selected for RCTs were mostly based on subjective perceptions, such as symptoms. It is difficult to assess the effects of RTX at a microscopic level without assessing certain biochemical markers associated with RNS. Finally, the tiny sample size makes it impossible to adequately examine the safety of RTX or other medications.

## 5. Conclusion

The results of this study suggest that RTX may be effective in RNS, as evidenced by remission rates and serum albumin. However, the effect on urinary protein was not significant. There is a lack of high-quality evidence in the relevant literature. Therefore, large sample, multicenter, low risk of bias clinical studies, as well as basic medical research, is needed.

## Figures and Tables

**Figure 1:** The inclusion process of literature.

**Figure 2:** Forest plot of the remission rate.

**Figure 3:** Remission rate sensitivity analysis for each study included in the review.

**Figure 4:** Forest plot of the remission rate after excluding one trail.

**Figure 5:** Forest plot of the serum albumin.

**Figure 6:** Forest plot of the urine protein.

**Figure 7:** Funnel plot of the remission rate.

**Table 1:** The main characteristics of the studies that were considered. NR: not reported; T: trial group; C: control group.

Study (ref.)	Country	Number of participants		Age (years) (mean ± SD)		Course of disease(years) (mean ± SD)		Rituximab dose	Follow-up time (month)
		T	C	T	C	T	C		
Dahan et al. [15]	France	37	38	53.0 ± 14.1	58.5 ± 14.3	NR	NR	375 mg/m^2^, 1 or 2 times a week	17
Ahn et al. [16]	South Korea	35	16	13.5 ± 5.0	12.5 ± 4.2	8.7 ± 4.9	7.4 ± 4.9	375 mg/m^2^, 1 time a week	12
Ravani et al. [17]	Italy	15	15	6.9 ± 3.6	6.9 ± 3.1	2.7 ± 2.4	2.0 ± 2.5	375 mg/m^2^	22
Ravani et al. [18]	Italy	27	27	10.2 ± 4.0	11.3 ± 4.3	5.7 ± 3.5	7.8 ± 4.0	375 mg/m^2^, 1 or 2 times a week	12
Basu et al. [19]	India	60	60	7.1 ± 2.8	7.2 ± 2.8	2.3 ± 1.7	2.5 ± 1.5	375 mg/m^2^, 1 time a week	12
Iijima et al. [20]	Japan	24	24	11.5 ± 5.0	13.6 ± 6.9	7.9 ± 4.7	8.0 ± 5.4	375 mg/m^2^, 1 time a week	12
Yao et al. [21]	China	25	25	37.6 ± 10.3	37.5 ± 10.3	21.53 ± 6.30	21.51 ± 6.27	375 mg/m^2^, 1 time a week	NA
Magnasco et al. [22]	Italy	16	15	8.5 ± 4.4	7.3 ± 3.7	2.5	1.4	375 mg/m^2^, 2 times a week	18

## Data Availability

The data could be obtained from contacting the corresponding author.

## References

[1] Radhakrishnan J., Cattran D. C. (2012). The KDIGO practice guideline on glomerulonephritis: reading between the (guide)lines—application to the individual patient. *Kidney International*.

[2] Boute N., Gribouval O., Roselli S. (2000). *NPHS2* encoding the glomerular protein podocin, is mutated in autosomal recessive steroid-resistant nephrotic syndrome. *Nature Genetics*.

[3] Tryggvason K., Wartiovaara J. (2001). Molecular basis of glomerular permselectivity. *Current Opinion in Nephrology and Hypertension*.

[4] Wen J., Chen X., Wei S., Ma X., Zhao Y. (2022). Research progress and treatment status of liver cirrhosis with hypoproteinemia. *Evidence-based Complementary and Alternative Medicine*.

[5] Chiu M. C. (2008). Management strategy for idiopathic nehprotic syndrome in children. *Zhong Nan Da Xue Xue Bao. Yi Xue Ban*.

[6] McAdams A. J., Valentini R. P., Welch T. R. (1997). The nonspecificity of focal segmental glomerulosclerosis. The defining characteristics of primary focal glomerulosclerosis, mesangial proliferation, and minimal change. *Medicine*.

[7] Uffing A., Hullekes F., Hesselink D. A. (2022). Long-term apheresis in the management of patients with recurrent focal segmental glomerulosclerosis after kidney transplantation. *Kidney International Reports*.

[8] Korbet S. M., Schwartz M. M., Lewis E. J. (2022). Primary focal segmental glomerulosclerosis: clinical course and response to therapy. *American Journal of Kidney Diseases*.

[9] McEnery P. T., Strife C. F. (1982). Nephrotic syndrome in childhood: management and treatment in patients with minimal change disease, mesangial proliferation, or focal glomerulosclerosis. *Pediatric Clinics of North America*.

[10] (1981). Primary nephrotic syndrome in children: clinical significance of histopathologic variants of minimal change and of diffuse mesangial hypercellularity. *Kidney International*.

[11] Kyrieleis H. A., Löwik M. M., Pronk I. (2009). Long-term outcome of biopsy-proven, frequently relapsing minimal-change nephrotic syndrome in children. *Clinical Journal of the American Society of Nephrology*.

[12] Ghiggeri G. M., Catarsi P., Scolari F. (2004). Cyclosporine in patients with steroid-resistant nephrotic syndrome: an open- label, nonrandomized, retrospective study. *Clinical Therapeutics*.

[13] Jayne D. (2010). Role of rituximab therapy in glomerulonephritis. *Journal of the American Society of Nephrology*.

[14] Benz K., Dötsch J., Rascher W., Stachel D. (2004). Change of the course of steroid-dependent nephrotic syndrome after rituximab therapy. *Pediatric Nephrology*.

[15] Dahan K., Debiec H., Plaisier E. (2017). Rituximab for severe membranous nephropathy: a 6-month trial with extended follow-up. *Journal of the American Society of Nephrology*.

[16] Ahn Y. H., Kim S. H., Han K. H. (2018). Efficacy and safety of rituximab in childhood-onset, difficult-to-treat nephrotic syndrome: a multicenter open-label trial in Korea. *Medicine (Baltimore)*.

[17] Ravani P., Rossi R., Bonanni A. (2015). Rituximab in children with steroid-dependent nephrotic syndrome: a multicenter, open-label, noninferiority, randomized controlled trial. *Journal of the American Society of Nephrology*.

[18] Ravani P., Magnasco A., Edefonti A. (2011). Short-term effects of rituximab in children with steroid- and calcineurin-dependent nephrotic syndrome: a randomized controlled trial. *Clinical Journal of the American Society of Nephrology*.

[19] Basu B., Sander A., Roy B. (2018). Efficacy of rituximab vs tacrolimus in pediatric corticosteroid-dependent nephrotic syndrome. *JAMA Pediatrics*.

[20] Iijima K., Sako M., Nozu K. (2014). Rituximab for childhood-onset, complicated, frequently relapsing nephrotic syndrome or steroid-dependent nephrotic syndrome: a multicentre, double-blind, randomised, placebo-controlled trial. *Lancet*.

[21] Fengliang Y., Junfei Q., Sisi Y. (2020). Clinical analysis of rituximab combined with hormone sequential therapy in the treatment of refractory microscopic nephrotic syndrome. *Modern Practical Medicine*.

[22] Magnasco A., Ravani P., Edefonti A. (2012). Rituximab in children with resistant idiopathic nephrotic syndrome. *Journal of the American Society of Nephrology*.

[23] Shalhoub R. J. (1974). Pathogenesis of lipoid nephrosis: a disorder of T-cell function. *Lancet*.

[24] Chan O. T., Hannum L. G., Haberman A. M., Madaio M. P., Shlomchik M. J. (1999). A novel mouse with B cells but lacking serum antibody reveals an antibody-independent role for B cells in murine lupus. *The Journal of Experimental Medicine*.

[25] Sfikakis P. P., Boletis J. N., Lionaki S. (2005). Remission of proliferative lupus nephritis following B cell depletion therapy is preceded by down-regulation of the T cell costimulatory molecule CD40 ligand: an open-label trial. *Arthritis and Rheumatism*.

